The article "lncRNA ABHD11‐AS1, regulated by the EGFR pathway, contributes to the ovarian cancer tumorigenesis by epigenetically suppressing TIMP2" was retracted in 2024. Reasons: duplicated images; overlap with earlier publications; signs of a paper mill; original data or images not available.

# lncRNA ABHD11‐AS1, regulated by the EGFR pathway, contributes to the ovarian cancer tumorigenesis by epigenetically suppressing TIMP2

**DOI:** 10.1002/cam4.2586

**Published:** 2019-09-30

**Authors:** Xiang‐Yang Zeng, Xiao‐Yan Jiang, Jia‐Hui Yong, Hui Xie, Jing Yuan, Da Zeng, Ying‐Yu Dou, Song‐Shu Xiao

**Affiliations:** ^1^ Department of Gynecology The Third Xiangya Hospital of Central South University Changsha P.R. China

**Keywords:** ABHD11‐AS1, EGFR, epithelial ovarian cancer, EZH2, TIMP2

## Abstract

**Objective:**

Epithelial ovarian cancer (EOC) is a common gynecologic malignancy characterized by extensive peritoneal metastasis and high mortality rate. ABHD11 Antisense RNA1 (ABHD11‐AS1) has recently been identified as a regulator of growth and metastasis in multiple tumors, including EOC. However, the biological function and potential mechanism of ABHD11‐AS1 in EOC remains poorly understood.

**Methods:**

Immunohistochemistry, western blot, and qRT‐PCR analysis were used to determine the expression pattern of ABHD11‐AS1 and epidermal growth factor receptor (EGFR) in both EOC tissues and cell lines, respectively. Colony formation, transwell and wound healing assays were performed to evaluate the roles of EGFR and ABHD11‐AS1 on the capacity of cell proliferation, migration, and invasion. Western blot analysis was performed to measure the regulation of EGFR pathway on STAT3. Moreover, chromatin immunoprecipitation was employed to demonstrate the interaction between ABHD11‐AS1 and STAT3. RNA immunoprecipitation was subjected to prove the direct binding between ABHD11‐AS1 and EZH2. Immunofluorescence staining was performed to measure the expression and localization of TIMP2. EOC mouse model was conducted for validating the role of ABHD11‐AS1 in vivo.

**Results:**

EGFR and ABHD11‐AS1 were highly expressed in EOC tissues and cell lines. Knockdown of EGFR or ABHD11‐AS1 inhibited cell growth, migration, and invasion of EOC cells. Expression of ABHD11‐AS1 was regulated by the activation of EGFR signaling pathway, mediated by STAT3. Besides, ABHD11‐AS1 was shown to silence TIMP2 by binding to chromatin‐modifying enzyme EZH2. Furthermore, inhibition of EGFR pathway or ABHD11‐AS1 repressed the tumor growth of EOC.

**Conclusion:**

We defined the regulatory relationship between the EGFR signaling pathway, ABHD11‐AS1, EZH2, and TIMP2 suggesting that ABHD11‐AS1 may act as an oncogene and a potential target for antitumor therapies in ovarian cancer.

## Graphical abstract

EGFR and NEAT1 are upregulated in epithelial ovarian cancer. EGFR and NEAT1 promote proliferation, migration, and invasion of ovarian cancer cells. NEAT1 is upregulated by activation of EGFR signaling pathway.

The article "lncRNA ABHD11‐AS1, regulated by the EGFR pathway, contributes to the ovarian cancer tumorigenesis by epigenetically suppressing TIMP2" was retracted in 2024. Reasons: duplicated images; overlap with earlier publications; signs of a paper mill; original data or images not available.

## 1 INTRODUCTION

Ovarian cancer, which is associated with high mortality rate, represents one of the most common gynecologic malignancy worldwide.^1^, ^2^ Epithelial ovarian cancer (EOC) accounts for approximately 90% of all ovarian cancer cases.^3^ Due to the lack of specific symptoms and effective screening method in early stage EOC (stages I and II), most patients are diagnosed with advanced EOC (stages III and IV).^4^ Despite recent advances in chemotherapy and cyto‐reductive surgery, the prognosis of EOC remains poor and the 5‐year survival rate of EOC patients is only 30%.^5^ EOC is characterized by extensive peritoneal metastasis, which is the leading cause of death.^6^ However, the specific molecular mechanism of extensive peritoneal metastasis in EOC remains elusive, and further investigation is needed.

The epidermal growth factor receptor (EGFR) belongs to the ErbB family of receptor tyrosine kinases. Mutations that upregulate EGFR are known to be linked to the development of a broad variety of tumors.^7^ These somatic mutations results in constant activation of EGFR and uncontrolled cell division. Antitumor therapeutics that target EGFR signaling has been developed, including gefitinib, erlotinib, and icotinib.^8^ High expression of EGFR is known to positively correlate with growth and progression of ovarian cancers, leading to poor prognosis in women with advanced cases.^9^

Long noncoding RNAs (lncRNAs) are nonprotein coding transcripts that are longer than 200 nucleotides.^10^, ^11^ Recent research suggest that dysregulation of lncRNAs is frequently identified in diverse varieties of cancers and plays pivotal roles in regulation of tumor growth and metastasis.^12^, ^13^ ABHD11 Antisense RNA1(ABHD11‐AS1), located at the human chromosome 7 q11.23, has been identified as an oncogene in multiple cancers. Upregulated ABHD11‐AS1 has been found in various types of tumors, including endometrial carcinoma, bladder cancer, colorectal cancer, and gastric cancer.^14^ Moreover, recent study has been demonstrated that ABHD11‐AS1 is upregulated in ovarian cancer and promotes the tumorigenesis and progression of ovarian cancer.^15^, ^16^ Another recent work on papillary thyroid carcinoma revealed that the transcriptional activity of ABHD11‐AS1 is regulated by STAT3 signaling pathway.^17^ However, available information on the roles of ABHD11‐AS1 in ovarian cancer is limited and further exploration is required.

Matrix metalloproteinases (MMPs) promote tumor cell invasion by degrading extracellular matrix (ECM), which is of major mechanisms of metastasis initiation. Tissue inhibitors of metalloproteinases (TIMPs) are endogenous regulators of MMPs that inhibit MMPs activity by binding to their active sites or sequestering the pro‐MMP zymogens. TIMPs exert suppressive functions on tumor metastasis, of which are downregulated in many solid tumors. There are four identified TIMPs: TIMP1, TIMP2, TIMP3, and TIMP4. Among them, Yi et al found the high expression of enhancer of zeste homolog 2 (EZH2) in ovarian cancer and its correlation with metastasis and poor patient survival, repressing TIMP2 expression via H3K27me3 and methylation. However, the role of TIMP2 in EOC remains little known.

The article "lncRNA ABHD11‐AS1, regulated by the EGFR pathway, contributes to the ovarian cancer tumorigenesis by epigenetically suppressing TIMP2" was retracted in 2024. Reasons: duplicated images; overlap with earlier publications; signs of a paper mill; original data or images not available.

In the present study, we aim to delineate the mechanism by which lncRNA ABHD11‐AS1 regulates growth and invasion of ovarian cancer with both in vitro and in vivo experiments. Our findings revealed that upregulation of ABHD11‐AS1 in ovarian cancer could be induced by the activation of EGFR signaling pathway. Subsequently, ABHD11‐AS1 epigenetically suppressed TIMP2 expression via binding to EZH2, which promotes invasion and metastasis of ovarian cancer. Thus, our data could further regard ABHD11‐AS1 as an oncogene and a potential target for antitumor therapeutics.

## 2 MATERIALS AND METHODS

### 2.1 Clinical sample collection

All experiments conducted in this study were approved by the Ethics Committee of the Third Xiangya Hospital of Central South University. All patients recruited to this study did not receive any preoperative treatment. Written informed consent was obtained from all patients. A cohort of 53 EOC tissues and adjacent nontumor ovarian tissues were collected from patients who underwent surgery at the Third Xiangya Hospital of Central South University. Collected tissues were washed with sterile phosphate‐buffered saline, immediately frozen in liquid nitrogen, and stored at −80°C. All diagnoses of EOC were confirmed by histology.

### 2.2 Cell culture and cell transfection

EOC cell lines (HO8910, OVCA429) and normal ovarian epithelial cell line (IOSE80) were obtained from American Type Culture Collection (ATCC). Cells were cultured at 37°C in a humidified incubator with 5% CO_2_. DMEM was used with 10% fetal bovine serum, 100 μg/mL streptomycin, and 100 U/mL penicillin.

Cells were transfected with shRNAs targeting ABHD11‐AS1, EGFR, or random scrambled shRNA control (purchased from GenePharma) using Lipofectamine 2000 transfection reagent (Invitrogen) according to the manufacturer instructions. EZH2 was silenced with siRNAs targeting EZH2 or scrambled siRNA control (purchased from GenePharma). Cells were harvested for further exploration 48 hours after transfection.

### 2.3 Immunohistochemistry

Ovarian cancer tissues were fixed in 4% paraformaldehyde, dehydrated, embedded in paraffin wax, and then cut into 5 µm sections. Slides were treated with xylene followed by ethanol, then rehydrated in distilled water. Sample was incubated with proteinase K for 30 minutes to allow antigen retrieval. Endogenous peroxidase activities were blocked by treatment with 0.3% hydrogen peroxide for 30 minutes. Nonspecific binding was blocked with 0.3% bovine serum albumin for 30 minutes. Slides were incubated with the primary antibody at 4°C overnight. Monoclonal antibodies for EGFR (Cell Signaling Technology, 1:100) and EZH2 (Cell Signaling Technology, 1:200) were used with 0.3% bovine serum albumin.

The article "lncRNA ABHD11‐AS1, regulated by the EGFR pathway, contributes to the ovarian cancer tumorigenesis by epigenetically suppressing TIMP2" was retracted in 2024. Reasons: duplicated images; overlap with earlier publications; signs of a paper mill; original data or images not available.

### 2.4 Total RNA extraction and real‐time PCR

Total cellular RNA was extracted from cancer tissues and cell lines with Trizol reagent (Invitrogen) following the manufacturer's instructions. Then the cDNA was synthesized with the Prime‐Script RT‐PCR master mix (Takara). For the quantitative RT‐PCR analysis, the cDNA was subjected to RT‐PCR using SYBR Green Premix Ex Taq (Takara) following the manufacturer's instructions. Each experiment was performed in duplicates and was repeated three times. The primers used for qRT‐PCR were as follows: EGFR (forward: 5′‐CCTATGTGCAGAGGAATTATGATCTTT‐3′ and reverse: 5′‐CCACTGTGTTGAGGGCAATG‐3′), ABHD11‐AS1 (forward: 5′‐TCCAGACAAGACTTGGTCGC‐3′ and reverse: 5′‐CAGCTGGTTGTGTGGCTTTC‐3′), STAT3 (5′‐CTCTTC GGGATGACAGGAGC‐3′ and reverse: 5′‐CTTGGGCGACGGTTT GAATC‐3′), TIMP2 (5′‐GCCAAAGCGTCAGTGAGA‐3′ and reverse: 5′‐AACGCTTCACGAATTTGCGT‐3′), GAPDH (5′‐AACAGGAGGTCCCTACTCCC‐3′ and reverse: 5′‐GCCATTTTGCGGTGGAAATG‐3′), and U6 (5′‐GCAGACCGTTCGTCAACCTA‐3′ and reverse: 5′‐AATTCTGTTTGCGGTGCGTC‐3′).

### 2.5 Colony formation assay

Human EOC cells (HO8910 and OVCA429) were trypsinzed at 80%‐90% confluence, pelleted, resuspended, and counted. Cells were transfected with shRNAs specifically targeting ABHD11‐AS1, EGFR, and their random scrambled shRNA. The cells were seeded with a density of 500 cells/well in 6‐well plates and incubated for 2 weeks for the colony formation assay. Cells were then washed with PBS, fixed with 10% formalin, stained with 0.5% crystal violet (Sigma) and finally counted.

### 2.6 Transwell assays

Transwell migration and invasion assay was performed with Boyden chambers carrying 8 μm pore membranes coated with Matrigel. Cells transfected with shRNA were seeded into the upper chamber with serum‐free DMEM. The lower chamber was filled with DMEM supplemented by 10% fetal bovine serum. After incubating for 24 hours, the remaining cells on the upper surface of the filter were collected with cotton swabs. The cells that have migrated the bottom of the top chamber were fixed with methanol and stained with 0.1% crystal violet for 10 minutes. The filters were then washed in PBS and observed under a light microscope.

The article "lncRNA ABHD11‐AS1, regulated by the EGFR pathway, contributes to the ovarian cancer tumorigenesis by epigenetically suppressing TIMP2" was retracted in 2024. Reasons: duplicated images; overlap with earlier publications; signs of a paper mill; original data or images not available.

### 2.7 Wound healing assay

Cells were seeded in 6‐well plates. Scratch wounds were made by scraping the cells layer across each well when the cell confluence reached about 80%. After wounding, the debris was washed by PBS. The migration of cells at the edge of the scratch was observed and captured under microscopy at indicated hours.

### 2.8 Total cell protein extraction and Western blot

EOC cells (HO8910 and OVCA429) were lysed with cold lysis buffer (RIPA buffer, 89900, Thermo Fisher), proteins were extracted from the lysates, and protein concentrations were quantified. Next, equal amounts of proteins from each group were purified with 10% SDS‐polyacrylamide gels and were transferred to a polyvinylidene difluoride membrane. Nonspecific binding was blocked by incubation with 5% skim milk for 1 hour. Next, the membrane was incubated with primary antibodies overnight at 4°C. Antibodies against EGFR, p‐EGFR, Snail, Slug, E‐cadherin, STAT‐3, pSTAT3, TIMP2, and EZH2 were purchased from Cell Signaling Technology (1:1000). Antibody against GAPDH was purchased from Proteintech (1:5000). The membrane was then treated with horseradish peroxidase‐conjugated secondary antibody for 1 hour. Then the antibody‐reactive bands were detected with the ECL reagent (Millipore Corp.).

### 2.9 CHIP detection

Chromatin immunoprecipitation (CHIP) experiments were performed with the EZ‐Magna ChIP kit. Ovarian cancer cells (HO8910 and OVCA429) were cross‐linked with 1% formaldehyde for 10 minutes at room temperature to allow formation of protein‐DNA crosslinks. Cells were then lysed and sonicated in lysis buffer to afford chromatin fragments. Next, the resulting fragments were extracted based on manufacturer's protocol.

### 2.10 RIP detection

RNA immunoprecipitation (RIP) experiments were performed with the Magna RIP RNA‐binding protein immunoprecipitation Kit according to the manufacturer's instructions. lncRNAs HOTAIR and MALAT1, which are known to bind to EZH2, were used for positive control groups. Lysates from EOC cell lines (HO8910 and OVCA429) were incubated with rabbit anti‐EZH2 (1:50) for 4 hours at 4°C. The resulting co‐precipitated RNAs were analyzed by qRT‐PCR.

### 2.11 Immunofluorescence

EOC cell lines (HO8910, OVCA429) were transfected with shABHD11‐AS1 or scrambled negative control RNA. Antibodies against TIMP2 and secondary antibodies with Alexa Fluor® 594 (1:1000, Life Technologies) were used for immunofluorescence staining. DAPI was used as a control for staining the nucleus. The FV‐1200 laser scanning confocal microscope was used for visualization.

The article "lncRNA ABHD11‐AS1, regulated by the EGFR pathway, contributes to the ovarian cancer tumorigenesis by epigenetically suppressing TIMP2" was retracted in 2024. Reasons: duplicated images; overlap with earlier publications; signs of a paper mill; original data or images not available.

### 2.12 Animal model of ovarian cancer peritoneal metastasis

Nude mice model of EOC was constructed by intraperitoneal injection of ovarian cancer cells. After successful model construction, EGFR inhibitor Gefitinib (100 mg/kg) or shABHD11‐AS1 was injected intraperitoneally twice a week over 5 weeks. Tumor size was measured with caliper after the animals were sacrificed. Tumor volume was measured every 5 days over 30 days to provide tumor growth curve.

### 2.13 Statistical analysis

Statistical analysis was performed with SPSS 16.0 (SPSS Inc). Student's *t* test was used to evaluate the differences between two groups. One‐way ANOVA was used to determine the differences among multiple groups. *P* values lesser than .05 (*P* < .05*) were considered as statistically significant; *P* values lesser than .01 (*P* < .01**) were considered as statistically highly significant.

## 3 RESULTS

### 3.1 Expression of EGFR and lncRNA ABHD11‐AS1 is upregulated in ovarian cancer

To explore the roles of EGFR and lncRNA ABHD11‐AS1, we firstly examined their expression levels both in EOC tissues and cell lines. Immunohistochemistry revealed markedly higher level of EGFR in EOC tissues compared with that of controls (Figure 1A), of which subcellular location is in the cell membrane and cytoplasm. Besides, qRT‐PCR and western blot analysis were employed and the results showed that EGFR and ABHD11‐AS1 were significantly upregulated in ovarian cancer tissues compared with normal tissues (Figure 1B,C). Moreover, EOC cell lines (OVCA429 and HO8910) and normal ovarian epithelial cell line (IOSE80) were recruited for further verification. Similarly, the level of EGFR and ABHD11‐AS1 also presented a higher expression in EOC cells compared to normal ovarian epithelial cells (Figure 1D,E). Therefore, these data implied that the aberrant upregulation of EGFR and ABHD11‐AS1 might participate in the progression of ovarian cancer.

**Figure 1:** The expression pattern of EFGR and ABHD11‐AS1 in ovarian cancer. A, Immunohistochemistry was used to detect EGFR expression levels in clinical cancer tissues and normal tissues. Scale bar, 300 μm. B, The expression of EGFR and ABHD11‐AS1 in ovarian cancer tissues was examined by qRT‐PCR. C, Expression of EGFR was examined in cancer tissues and in normal tissues by western blot. GAPDH was used as control. D, qRT‐PCR was performed to measure expression of EGFR and ABHD11‐AS1 in EOC cells (OVCA429 and HO8910) and normal ovarian epithelial cells (IOSE80). E, Western blot was used to examine expression of EGFR in EOC cell lines and in normal epithelial cells. GAPDH was used as control. *P < .05, **P < .01

### 3.2 EGFR and ABHD11‐AS1 promote proliferation, migration, and invasion of ovarian cancer cells

To investigate the effects of EGFR and ABHD11‐AS1 on cancer cells' biological functions, the following experiments were performed. We induced knockdown of EGFR or ABHD11‐AS1 in ovarian cancer cell lines with the corresponding shRNAs. Colony formation assay was employed to detect cell proliferation and the results showed that compared with the negative control group, significant reduction of colony numbers was observed in both EGFR and ABHD11‐AS1 knockdown groups (Figure 2A). Moreover, we found that depletion of EGFR or ABHD11‐AS1 resulted in significant decreases in migration and invasion of OVCA429 and HO8910 cells (Figure 2B). In addition, the suppressive effects of EGFR or ABHD11‐AS1 knockdown on cell migration were also demonstrated using wound healing assay (Figure 2C). Besides, EOC is known to progress via the epithelial‐mesenchymal transition (EMT), during which cells lose cell‐cell adhesion, and develop migratory and invasive characteristics.^23^ Transcription factors Snail1 and Slug are known to downregulate adhesion molecule E‐cadherin and promote EMT.^24^, ^25^ Thus, the examination of EMT‐related markers was performed by western blot analysis and the results showed that Snail, Slug, and Vimentin were decreased, while E‐cadherin was increased after knockdown of EGFR or ABHD11‐AS1, consistent with inhibition of cancer cell migration and invasion (Figure 2D). Altogether, these data implied that EGFR or ABHD11‐AS1 might exert oncogenic functions in ovarian cancer.

The article "lncRNA ABHD11‐AS1, regulated by the EGFR pathway, contributes to the ovarian cancer tumorigenesis by epigenetically suppressing TIMP2" was retracted in 2024. Reasons: duplicated images; overlap with earlier publications; signs of a paper mill; original data or images not available.

**Figure 2:** Knockdown EGFR and ABHD11‐AS1 suppress proliferation, migration, and invasion of ovarian cancer cells. A, Colony formation assay was used to detect changes in proliferation properties of OVCA429 and HO8910 cells after knockdown of EGFR or ABHD11‐AS1. B, Transwell assay was performed to test cancer cell migration and invasion ability after knockdown of EGFR or ABHD11‐AS1. C, Wound healing assay was performed after knockdown of EGFR or ABHD11‐AS1. D, Western blot was used to measure expression levels of epithelial‐mesenchymal transition (EMT)‐related proteins (Snail, Slug, E‐cadherin, and Vimentin). GAPDH was used as loading control. *P < .05, **P < .01

### 3.3 Activation of the EGFR signaling pathway stimulates lncRNA ABHD11‐AS1 via STAT3

To further explore the correlation between EGFR and ABHD11‐AS1, we overexpressed or silenced EGFR expression in both OVCA429 and HO8910 cells. As shown in Figure 3A, EGFR and p‐EGFR (the only activated form of EGFR) were both markedly upregulated in cells overexpressing EGFR and downregulated in cells silencing EGFR. Besides, qRT‐PCR analysis also indicated the positive correlation between EGFR and ABHD11‐AS1 (Figure 3B). In addition, the application of EGF dramatically induced the upregulation of p‐EGFR and EGFR and increased ABHD11‐AS1 expression (Figure 3C,D). Transcription factor STAT3 is known to act downstream of the EGFR pathway, and activated by its phosphorylation.^17^, ^26^, ^27^ Similarly, we found that knockdown of EGFR restrained the level of p‐STAT3, while overexpression of EGFR promoted the activation of STAT3 (Figure 3E). Moreover, the level of p‐STAT3 can be induced by EGF stimulation (Figure 3F). These results implied that STAT3 may be as a downstream target of EGFR pathway. Furthermore, CHIP assay was performed and revealed that STAT3 directly bound to the promoter of ABHD11‐AS1 modulating the transcriptional activity of ABHD11‐AS1(Figure 3G). Meanwhile, ABHD11‐AS1 level was significantly reduced once knockdown of STAT3 (Figure 3H). Therefore, our findings suggested that ABHD11‐AS1 might be regulated by the EGFR signaling pathway through activation of STAT3.

The article "lncRNA ABHD11‐AS1, regulated by the EGFR pathway, contributes to the ovarian cancer tumorigenesis by epigenetically suppressing TIMP2" was retracted in 2024. Reasons: duplicated images; overlap with earlier publications; signs of a paper mill; original data or images not available.

**Figure 3:** Activation of EGFR signaling pathway induces lncRNA ABHD11‐AS1 expression. A, Western blot was used to confirm that EGFR and p‐EGFR expression were tuned by knockdown or overexpression. B, Expression of ABHD11‐AS1 after knockdown or overexpression of EGFR was measured by qRT‐PCR. C, Western blot was used to examine expression levels of p‐EGFR and EGFR in OVCA429 and HO8910 cell lines after EGF stimulation. GAPDH was used as loading control. D, Expression of ABHD11‐AS1 was measured by qRT‐PCR with EGF treatment. E and F, Western blot was used to examine the expression levels of STAT3 and their respective phosphorylation levels. GAPDH was used as loading control. G, Chromatin immunoprecipitation (CHIP) was performed to investigate the interactions between transcription factors STAT3 and the promoter region of ABHD11‐AS1. H, qRT‐PCR was used for validation of STAT3 and ABHD11‐AS1 expression after silencing STAT3. *P < .05, **P < .01

### 3.4 lncRNA ABHD11‐AS1 promotes ovarian cancer tumorigenesis by repression of TIMP2

TIMP2 is regarded as a repressor of tumor, of which downregulation is observed in many solid tumors, including ovarian cancer. However, whether TIMP2 gets involved in ABHD11‐AS1‐mediated biological functions in ovarian cancer remains little known. Subsequently, the level of TIMP2 was found to be lower in EOC cells (OVCA429 and H08910), comparing to normal ovarian epithelial cells (IOSE80) (Figure 4A). To investigate the correlation between ABHD11‐AS1 and TIMP2, qRT‐PCR assay was performed and the results showed that knockdown of ABHD11‐AS1 significantly increased the expression of TIMP2 (Figure 4B), Moreover, the expression of TIMP2 in both OVCA429 and HO8910 cells was significantly increased after ABHD11‐AS1 knockdown (Figure 4C). To address if TIMP2 is a functional downstream target of ABHD11‐AS1 in ovarian cancer, TIMP2 was silenced in ABHD11‐AS1 knocking down cells. As expected, silencing TIMP2 dramatically rescued lack of ABHD11‐AS1 resulted in the colony growth delay (Figure 4D). Moreover, silencing TIMP2 also markedly reversed the inhibition of migration and invasion induced by ABHD11‐AS1 knockdown (Figure 4E). Taken together, the data suggested that lncRNA ABHD11‐AS1 might exert its oncogenic functions through suppressing TIMP2, contributing to the progression of ovarian cancer.

The article "lncRNA ABHD11‐AS1, regulated by the EGFR pathway, contributes to the ovarian cancer tumorigenesis by epigenetically suppressing TIMP2" was retracted in 2024. Reasons: duplicated images; overlap with earlier publications; signs of a paper mill; original data or images not available.

**Figure 4:** lncRNA ABHD11‐AS1 knockdown inhibits ovarian cancer cell progress by TIMP2. A, TIMP2 expression was detected by qRT‐PCR in EOC cells (OVCA429 and HO8910) and normal ovarian epithelial cells (IOSE80). B, Western blot was used to examine the expression of TIMP2 after knockdown of ABHD11‐AS1. GAPDH was used as control. C, Immunofluorescence assay was employed to detect the visualization of TIMP2 in EOC cells. Scale bar, 200 μm. D, Colony formation assay was used to detect changes in proliferation properties of cancer cells (OVCA429 and HO8910) after knockdown of TIMP2 together with sh‐ABHD11‐AS1 compared with negative control or knockdown of ABHD11‐AS1 alone. E, Transwell assay was performed to observe cell migration and invasion in shNC, shABHD11‐AS1 alone, or shABHD11‐AS1 +siTIMP2 EOC cell lines. *P < .05, **P < .01

### 3.5 lncRNA ABHD11‐AS1 epigenetically suppresses TIMP2 via binding to EZH2

lncRNAs are known to interact with EZH2, the catalytic subunit of the epigenetic regulatory complex PRC2, to mediate expression of downstream genes.^28^, ^29^ To further explore the underlying mechanism of ABHD11‐AS1, RIP was subjected to detect the potential interaction between ABHD11‐AS1 and EZH2 in EOC cell lines. As shown in Figure 5A, ABHD11‐AS1 was found to bind EZH2 with comparable affinities as lncRNAs HOTAIR and MALAT1, which are known to bind to EZH2.^28^, ^29^ We also verified that silencing of EZH2 increased the expression of TIMP2 (Figure 5B). Moreover, CHIP assay demonstrated that shABHD11‐AS1 decreased the recruitment of H3K27me3 at the TIMP2 promoter (Figure 5C). Furthermore, after overexpression of ABHD11‐AS1, as expected, the expression of TIMP2 was downregulated. However, this effect was reversed by siEZH2 transfection (Figure 5D). Overall, lncRNA ABHD11‐AS1 might repress TIMP2 through EZH2‐mediated epigenetic modulation.

**Figure 5:** lncRNA ABHD11‐AS1 binds to EZH2 to epigenetically repress TIMP2. A, RNA immunoprecipitation was used to detect the binding relationship between ABHD11‐AS1 and EZH2. HOTAIR and MALAT1 were used as positive controls. B, Western blot was used to examine the TIMP2 expression of after knockdown of EZH2. GAPDH was used as control. C, qRT‐PCR analysis of immunoprecipitated chromatin by H3K27me3 antibody on TIMP2 promoter. IgG served as a negative control. D, Western blot was used to detect expression of TIMP2. GAPDH was used as loading control. *P < .05, **P < .01

The article "lncRNA ABHD11‐AS1, regulated by the EGFR pathway, contributes to the ovarian cancer tumorigenesis by epigenetically suppressing TIMP2" was retracted in 2024. Reasons: duplicated images; overlap with earlier publications; signs of a paper mill; original data or images not available.

### 3.6 Inhibition of EGFR or ABHD11‐AS1 impedes tumor growth in vivo

We further validated the role of EGFR and ABHD11‐AS1 in vivo. A mouse model of ovarian cancer was constructed via intraperitoneal injection of cancer cells for further confirmation. EGFR inhibitor Gefitinib or shABHD11‐AS1 was injected intraperitoneally twice a week over 5 weeks. Compared with model mice without any treatment, we found significant reduction in tumor sizes in the mice treated with Gefitinib or shABHD11‐AS1 (Figure 6A). Compared with the model group, tumor growth was significantly slowed and inhibited in the Gefitinib treated or shABHD11‐AS1‐treated groups (Figure 6B). Tumor weights were markedly lower with Gefitinib or shABHD11‐AS1 treatment compared with no treatment (Figure 6C). Besides, immunohistochemistry was performed to examine the expression of EZH2 and the results showed that EZH2 was markedly inhibited in groups treated with Gefitinib or shABHD11‐AS1 (Figure 6D). We also observed a significant decrease in both EZH2 and ABHD11‐AS1 expression when the model mice were administered Gefitinib or shABHD11‐AS1 (Figure 6E). In addition, the expression of TIMP2 was clearly accumulated after Gefitinib treatment or shABHD11‐AS1 (Figure 6F). These data indicated that EGFR/ABHD11‐AS1/TIMP2 axis might be involved in the tumorigenesis of ovarian cancer, providing a potential strategy for antitumor therapies.

**Figure 6:** EGFR regulated‐ABHD11‐AS1 in the progression of ovarian cancer progress in vivo. A, Comparison of tumor sizes between groups treated with Gefitinib, with shABHD11‐AS1, and no treatment. B, Tumor growth curve for groups treated with Gefitinib, with shABHD11‐AS1, and no treatment. C, Tumor weight for groups treated with Gefitinib, with shABHD11‐AS1, and no treatment. D, Immunohistochemistry was used to detect expression of EZH2 in groups treated with Gefitinib, with shABHD11‐AS1, and no treatment. Scale bar, 300 μm. E, qRT‐PCR was used to examine the expression of ABHD11‐AS1 and EZH2 in groups treated with Gefitinib, with shABHD11‐AS1, and no treatment. F, Western blot was used to detect the expression of EZH2 and TIMP2 in groups treated with Gefitinib, with shABHD11‐AS1, and no treatment. GAPDH was served as loading control. *P < .05, **P < .01

The article "lncRNA ABHD11‐AS1, regulated by the EGFR pathway, contributes to the ovarian cancer tumorigenesis by epigenetically suppressing TIMP2" was retracted in 2024. Reasons: duplicated images; overlap with earlier publications; signs of a paper mill; original data or images not available.

## 4 DISCUSSION

Metastasis of EOC is intricately related to its tumor microenvironment.^30^ The EGF/EGFR signaling pathway is known to play an important role in modulating the tumor microenvironment, and upregulation of the EGFR signaling pathway is associated with uncontrolled cell division and poor prognosis for multiple cancer types.^31^, ^32^ In the case of ovarian cancer, overexpression of EGFR has been linked with tumor growth and metastasis.^9^ However, the specific mechanism by which the EGFR pathway regulates the tumorigenesis of EOC remains poorly understood. In the present study, we examined expression of EGFR in EOC clinical cancer tissues and in EOC cell lines. The results revealed significantly higher expression of EGFR in cancer tissues/cell lines than in normal tissue/cell lines. We further found that knockdown of EGFR resulted in inhibition of proliferation, migration, and invasion of EOC cells. The inhibitory effect of EGFR knockdown on tumor growth was also confirmed in EOC mouse model. EGFR knockdown was also shown to cause inhibition of EMT, based on changes in expression levels of EMT‐associated factors. In summary, our study suggested that expression of EGFR is positively correlated with growth and invasion of EOC.

Aberrant expression of lncRNA ABHD11‐AS1 has been reported to be involved in regulating the development and progression of various tumors, including endometrial carcinoma, bladder cancer, colorectal cancer, and gastric cancer. Specifically for ovarian cancer, several recent studies have proved that high expression of ABHD11‐AS1 is positively associated with tumor growth and invasion.^15^, ^16^ Similarly, we also confirmed high expression of ABHD11‐AS1 in both EOC tissues and cell lines. Further functional researches verified that knockdown of ABHD11‐AS1 could notably repress cell proliferation, migration, and invasion of ovarian cancer cells. In addition, in vivo experiments further confirmed that ABHD11‐AS1 knockdown resulted in inhibition of tumor growth and reduction in tumor size. Herein, our study indicated the oncogenic functions of ABHD11‐AS1 in ovarian cancer. Meanwhile, we demonstrated the positive correlation of EGFR and ABHD11‐AS1 in EOC tissues. Further researches also verified that knockdown of EGFR resulted in decreased phosphorylation level for STAT3, which binds the promoter region of ABHD11‐AS1. Thus, our data implied that ABHD11‐AS1, regulated by EGFR pathway, contributes to the tumor growth and invasion of EOC.

Abnormal expression of TIMP2 has been implicated in growth and invasion of multiple malignant tumors.^18^ Several upstream factors have been reported to mediate tumor progression and metastasis through the TIMP2.^19^, ^20^, ^21^ For instance, EZH2 was found to promote metastasis via TIMP2 signaling pathway in EOC.^20^ However, the relationship between lncRNA ABHD11‐AS1 and TIMP2 has not been studied in detail. In the present work, we showed that knockdown of ABHD11‐AS1 resulted in increased expression of TIMP2, which are negative regulatory factors of MMPs. Previous computational prediction and biochemical experiments suggested that EZH2 may be a potential downstream binding target of ABHD11‐AS1.^17^, ^22^ Here, we showed by RIP that ABHD11‐AS1 binds EZH2 with comparable affinities as lncRNAs HOTAIR and MALAT1, which are known to bind to EZH2.^28^, ^29^ Therefore, we provided evidence that ABHD11‐AS1 regulates the TIMP2 expression by binding with EZH2.

The article "lncRNA ABHD11‐AS1, regulated by the EGFR pathway, contributes to the ovarian cancer tumorigenesis by epigenetically suppressing TIMP2" was retracted in 2024. Reasons: duplicated images; overlap with earlier publications; signs of a paper mill; original data or images not available.

Taken together, this work delineated an integrated axis consisting of the EGFR signaling pathway, ABHD11‐AS1, EZH2, and TIMP2 in EOC. We established that activation of the EGFR signaling pathway enhances the expression of ABHD11‐AS1, which in turn recruits EZH2 to silence TIMP2 expression, and mediates invasion and metastasis. This work lays the foundation for further mechanistic studies and for discovery of a novel in antitumor therapeutics.

## ACKNOWLEDGMENTS

This work is supported by the Project of Hunan Provincial Natural Science Foundation (Grant No. 2018JJ3782) and the New Xiangya Talent Project of the Third Xiangya Hosipital of Central South University (20160308).

## CONFLICT OF INTEREST

The authors declare that they have no conflict of interest.

## Data Availability

All data generated or analysed during this study are included in this published article.
